The article "Correlation between Drug Resistance of Klebsiella Pneumonia and Antimicrobial Drug Usage" was retracted in 2023. Reasons: signs of a paper mill; unreliable results or conclusions.

# Correlation between Drug Resistance of *Klebsiella Pneumonia* and Antimicrobial Drug Usage

**DOI:** 10.1155/2022/2691134

**Published:** 2022-05-09

**Authors:** Anyun Liu, Jun Dai, Ru Shen, Feng Zhong, Xuehe Sheng, Houbao Huang

**Affiliations:** The Second Affiliated Hospital of Wannan Medical College, No. 10 Kangfu Road, Wuhu City, Anhui Province, China

## Abstract

*Objective. *To assess the correlation between the drug resistance of *Klebsiella pneumoniae* and antimicrobial drug usage. *Methods*. The drug resistance rate of *Klebsiella pneumoniae* and the antimicrobial drug dosage of inpatients admitted to The Second Affiliated Hospital of Wannan Medical College from January 2016 to December 2020 were retrospectively recorded, and their correlation was analyzed using the Pearson method. *Results*. There are 6493 strains of Gram-negative bacteria, including 1272 strains of *Klebsiella pneumoniae*, ranking first in respiratory medicine. *Klebsiella pneumoniae* showed an overall increasing trend in resistance to piperacillin/tazobactam and ampicillin/sulbactam and a high resistance to aztreonam, ceftazidime, and ciprofloxacin (all *P* < 0.05). The top 3 antimicrobial drugs used in 2016–2020 were *β*-lactams, quinolones, and macrolides. The rates of resistance to piperacillin/tazobactam, cefoperazone/sulbactam, and ampicillin/sulbactam were highly positively correlated with the use of *β*-lactams. The use of carbapenems and glycopeptides was negatively correlated with the resistance to ciprofloxacin, and the resistance to ceftazidime had a high positive correlation with the use of glycopeptides and carbapenems. *Conclusion*. The use of antimicrobial drugs is correlated with the resistance rate of *Klebsiella pneumoniae*. To reduce bacterial drug resistance, the rational use of antimicrobial drugs requires joint control through multiple departments to improve the clinical use of antimicrobial drugs and improve in-hospital control.

## 1. Introduction

*Klebsiella pneumoniae* is the most important group of bacteria in the Enterobacteriaceae family (commonly known as *S. pneumoniae*) [1], which invades the lungs via the respiratory tract and causes lobar or lobular fusion solids [2]. It is a common opportunistic pathogen in clinical practice [3, 4] that causes infections in the respiratory system, abdominal cavity, and urinary tract, with a high morbidity and mortality rate. In recent years, the massive use of antimicrobial drugs has resulted in a serious multidrug resistance of *Klebsiella pneumoniae* to commonly used antimicrobials. As reported by the 2017 China Bacterial Resistance Surveillance Network, the resistance rates of *Klebsiella pneumoniae* to imipenem and meropenem increased from 3.0% and 2.9% in 2005 to 20.9% and 24.0% in 2017, respectively [5, 6]. Antibacterial agents refer to products obtained from microorganisms such as bacteria, actinomycetes, and fungi in culture and also include various antibiotics, sulfonamides, imidazoles, nitroimidazoles, quinolones, and other chemically synthesized drugs [7]. Antimicrobial drugs have inhibitory and killing effects on pathogens at certain concentrations and are widely used in clinical practice [8]. Related studies have shown that the relationship between the use of antimicrobial drugs and bacterial resistance may provide guidance for the use of antimicrobial drugs [9, 10]. Accordingly, this study analyzed the correlation between the use of antimicrobial drugs and the resistance of *Klebsiella pneumoniae* in hospitalized patients admitted to The Second Affiliated Hospital of Wannan Medical College from January 2016 to December 2020 to provide a reference for the management of antimicrobial drugs. The results are reported as follows.

## 2. Materials and Methods

### 2.1. Source of Strains

*Klebsiella pneumoniae* isolated from the sputum, urine, blood, and cerebrospinal fluid from hospitalized patients admitted to The Second Affiliated Hospital of Wannan Medical College from January 2016 to December 2020 were collected, excluding the same bacteria isolated repeatedly from the same patients. In the statistical analysis of drug resistance, cases of drug resistance caused by the combination of multiple drugs were excluded to avoid duplication of data. The isolated strains were cultured as per the National Clinical Laboratory Operating Procedures. The drug resistance data of the strains were summarized by year, and the drug sensitivity test and bacterial identification were performed by the VITEK2 automatic microbiological analysis system. This study was approved by the Ethics Committee of The Second Affiliated Hospital of Wannan Medical College, No. J187WN.

### 2.2. Drug Sensitivity Assay

The K-B diffusion method was used for the assay of drug sensitivity, and the results were determined as per the rules established by the National Committee for Clinical Laboratory Standardization (CLISI) in January 2002, M100.S12 edition, and analyzed using WHONET 5.3.

### 2.3. Calculation

The data on all antimicrobial drug usage in the inpatient department from 2016 to 2020 were obtained through the drug management software system of The Second Affiliated Hospital of Wannan Medical College. The Defined Daily Doses (DDDs) method recommended by the World Health Organization (WHO) was used to calculate the frequency of antimicrobial drug use (DDDs).

(1) $$\begin{array}{c} \text{DDDs}=\frac{\text{total dose }\left(\text{gram}\right)\text{ of a drug consumed in a certain period}}{\text{DDD value of the drug}}. \end{array}$$

The DDD values were calculated according to the values specified by WHO and the dose recommended by the drug instruction. Quality control strains including *Escherichia coli* (ATCC 25922, ATCC 35218) and *Klebsiella pneumoniae* (ATCC 700603) were purchased from Wenzhou Kangtai Biotechnology Co.

### 2.4. Statistical Analysis

GraphPad Prism 8 software was used to plot the images, SPSS 22.0 software was used for data analysis, and Pearson analysis was used for correlation analysis. Count data are expressed as (*n* (%)) and analyzed using the chi-square test, while the measurement data are expressed as (mean ± SD) and analyzed using the *t*-test. r > 0 means the two variables are positively correlated, and *r* < 0 means they are negatively correlated. 0 ≤ |r| < 0.5 indicates a weak correlation between the two variables, 0.5 ≤ |r| ≤ 0.8 indicates a moderate correlation between the two variables, and |r| > 0.8 indicates a high correlation between the two variables. Differences were considered statistically significant at *P* < 0.05.

## 3. Results

### 3.1. The Isolation Rate of *Klebsiella pneumoniae*

A total of 6493 strains of Gram-negative bacteria were isolated from all the eligible patients from 2016 to 2020, with 1272 strains of *Klebsiella pneumoniae* (19.59%). The strain isolation rates were approximately equal for each year (*P* < 0.05). (Table 1).

The top-ranked departments for detection of *Klebsiella pneumonia* were respiratory medicine, neurology, critical care medicine, and cardiovascular medicine (Figure 1).

### 3.2. Resistance Rates of *Klebsiella pneumonia*

*Klebsiella pneumoniae* showed an overall increasing trend in resistance to piperacillin/tazobactam and ampicillin/sulbactam (9.6–2.99–7.14–8.11–13.49, and 41.2–/–24.21–29.15–30.74) and a high resistance to ceftazidime, aztreonam, and ciprofloxacin (18.71–22.02–24.49–27.70–28.28, 19.98–15.13–19.73–18.24–23.10, and 22.37–12.84–19.05–27.03–33.79), fluctuating around 30.00 (all *P* < 0.05). (Table 2).

### 3.3. Antibacterial Drug Usage

From 2016 to 2020, *β*-lactams, quinolones, and macrolides (59.31, 17.69, and 10.59) ranked in the top three as the most used antimicrobial drugs. The usage of *β*-lactams, tetracyclines, quinolones, and lincomycin increased, while the usage of aminoglycosides decreased year by year. Fluctuations were observed in lincomycin, nitroimidazoles, carbapenem, macrolides, and glycopeptides but failed to establish a significant trend (Table 3).

### 3.4. Correlation between *Klebsiella pneumonia* Resistance Rate and Antimicrobial Drug Usage

The resistance to piperacillin/tazobactam, cefoperazone/sulbactam, and ampicillin/sulbactam was positively correlated with the use of *β*-lactams (*r* = 0.965, *r* = 0.971, *r* = 0.872, *P* < 0.05), the use of carbapenem and glycopeptides was negatively correlated with ciprofloxacin resistance, and the resistance to ceftazidime was positively correlated with the usage of glycopeptides and carbapenem (*r* = 0.865, *r* = 0.874, all *P* < 0.05). They were all highly correlated (Table 4).

## 4. Discussion

*Klebsiella pneumoniae* can cause infections in the respiratory system, abdominal cavity, urinary tract, surgical incisions, abdominal cavity, and even sepsis, with a high morbidity and mortality rate [11]. Studies have reported two types of *Klebsiella pneumonia*, namely, highly virulent *Klebsiella pneumonia* and classical *Klebsiella*, which have different pathogenicity and virulence, and highly virulent *Klebsiella pneumonia* is highly invasive [12, 13]. In recent years, the massive use of antimicrobial drugs and the emergence of highly virulent strains resistant to various antimicrobial drugs have posed a great challenge to clinical treatment [14, 15]. Antibacterial agents refer to the products obtained from bacteria, actinomycetes, fungi, and other microorganisms in culture or various antibiotics, sulfonamides, imidazoles, nitroimidazoles, quinolones, and other chemically synthesized drugs [16, 17]. It has been reported that antimicrobial drugs have inhibitory and killing effects on pathogens at certain concentrations and are widely used in clinical practice [18]. Relevant studies have demonstrated that the amount and frequency of antimicrobial drugs used have a considerable influence on bacterial resistance [19, 20]. In the present study, 6493 Gram-negative strains were isolated from all included patients, including 1272 strains of *Klebsiella pneumonia* (19.59%), with approximately equal isolation rates each year, and the top-ranked departments for the detection of *Klebsiella pneumonia* included respiratory medicine, neurology, intensive care medicine, and cardiovascular medicine. Most of the patients in these departments are critically ill, elderly, bedridden, and diabetic and received antimicrobial drugs with long treatment cycles, with frequent invasive operations such as tracheal intubation, catheterization, and ventilator use, which further indicates that *Klebsiella pneumoniae* is a conditionally pathogenic organism that causes opportunistic infections in people with immunocompromised function, malignant tumors, and preexisting health conditions. *Klebsiella pneumonia* showed an overall increasing trend in resistance to piperacillin/tazobactam, and ampicillin/sulbactam (9.6–2.99–7.14–8.11–13.49 and 41.2–/–24.21–29.15–30.74), and a high resistance to piperacillin, ceftazidime, aztreonam, and ciprofloxacin (18.71–22.02–24.49–27.70–28.28, 19.98–15.13–19.73–18.24–23.10, and 22.37–12.84–19.05–27.03–33.79), fluctuating around 30.00 (all *P* < 0.05). From 2016 to 2020, *β*-lactams, quinolones, and macrolides antibiotics (59.31, 17.69, and 10.59) ranked in the top three as the most used antimicrobial drugs. The usage of *β*-lactams, tetracyclines, quinolones, lincomycin, and nitroimidazoles increased, while the usage of aminoglycosides decreased year by year. Fluctuations were observed in carbapenem, macrolides, and glycopeptides but failed to establish a significant trend. Resistance to piperacillin/tazobactam, cefoperazone/sulbactam, and ampicillin/sulbactam was highly positively correlated with the use of *β*-lactams, the use of carbapenem and glycopeptides was negatively correlated with ciprofloxacin resistance, and the resistance to ceftazidime was highly positively correlated with the usage of glycopeptides and carbapenem. *β*-Lactams inhibitors are a good choice for anti-*Klebsiella pneumonia* and have become the preferred treatment in clinical practice. However, in recent years, the resistance to piperacillin/tazobactam, cefoperazone/sulbactam, and ampicillin/sulbactam in our hospital has been positively correlated with the use of *β*-lactams, and the elevated resistance may be attributed to their frequent use. The resistance to ceftazidime was positively correlated with the usage of glycopeptides and carbapenem, which was consistent with the results of previous research [21], and the high usage of antimicrobial drugs was one of the important causes of *Klebsiella pneumonia* resistance (all *P* < 0.05).

The main causes of antibiotic resistance in *Klebsiella pneumonia* include the production of inactivating or passivating enzymes, such as *β*-lactamases, and aminoglycoside passivating enzymes, impaired penetration of antibiotics, or inability of antibiotics to reach the target site of action to produce antibacterial efficacy due to active efflux pumps, chromosomal mutations, alterations in the target site of action of antibiotics due to resistant plasmids, and alterations in metabolic pathways. The main *β*-lactamases associated with *Klebsiella pneumoniae* are the chromosome-mediated cephalosporin hydrolase (Amp-C enzyme), plasmid-mediated TEM, and SHV enzymes and their derivatives, consisting of ultrabroad-spectrum B-lactamases (ESBLs), carbenzylpenicillinase, o-chloropenicillinase (OXA enzyme), and nonmetallic carbapenemases. The production of ESBLs among these *β*-lactamases is most important in *Klebsiella pneumoniae*.

A reasonable combination of Chinese and Western medicines can improve the efficacy and shorten the course of treatment, while their unreasonable combination is associated with pharmacological contraindications. The Chinese herbal medicines for clearing heat and detoxifying toxins are known as “green antibiotics.” Compared with western antibiotics, these Chinese medicines have fewer side effects and higher safety, without causing bacterial resistance while inhibiting and killing bacteria, and they also improve the efficacy of drug resistance to varying degrees. Traditional Chinese medicinal herbs such as Violae Herba, Isatidis root, Chinese Lobelia, and dandelion have antiinflammatory and antibacterial effects. In the case of restricted use of antibiotics, herbal treatment offers a backup option for the treatment of infectious diseases. Fructus Aurantii Immaturus combined with gentamicin potentiates the treatment efficacy of *Klebsiella pneumonia*, which is attributed to the ability of Fructus Aurantii Immaturus to significantly increase the concentration of gentamicin in the bile duct, thereby enhancing the antibacterial power of gentamicin. The combination of herbal medicines containing acidic components with tetracycline antibiotics increases their bactericidal effects and enhances their effectiveness.

## 5. Conclusion

The correlation between the use of certain antimicrobial drugs and the resistance of *Klebsiella pneumonia* suggests that multidepartmental efforts should be directed toward the joint control of the rational use of antimicrobial drugs to reduce bacterial resistance and improve the rational clinical use of antimicrobial drugs. Accordingly, this study proposes the following suggestions: (1) The Antimicrobial Stewardship-multidisciplinary team (AMS-MDT) was established to achieve the administrative control of antimicrobial drugs, and three technical support systems composed of infection physicians, clinical microbiology testers, and clinical pharmacists were developed to jointly discuss antiinfection protocols for drug-resistant bacteria from different specialties and multiple perspectives. (2) Training and assessment were strengthened to improve clinicians' awareness and level of rational use of antimicrobial drugs. (3) The system of bacterial drug resistance detection and clinical application evaluation of antimicrobial drugs was improved [10], and the antimicrobial drug catalog and management plan were adjusted regularly . (4) A sound hospital infection prevention and control system to minimize the spread of drug-resistant bacteria in hospitals was developed. The limitations of this study are that targeting studies and further studies on the molecular mechanisms of the drugs with the highest resistance rates were absent, which will be explored in future studies.

## Figures and Tables

**Figure 1:** Top-ranked departments in the detection of *Klebsiella pneumonia* between 2016 and 2020.

**Table 1:** *Klebsiella pneumoniae* isolation rate between 2016 and 2020 (%).

	2016	2017	2018	2019	2020	Total
Gram-negative bacteria	1058	1312	1264	1373	1486	6493
*Klebsiella pneumoniae*	160	218	302	299	293	1272
Isolation rate	15.12	16.62	23.89	21.78	19.72	19.59
*x* ^2^			6.145			
*P*			＜0.001			

**Table 2:** Resistance rates of *Klebsiella pneumoniae* between 2016 and 2020 (%).

Antibacterials	Years				
	2016	2017	2018	2019	2020
Amikacin	2.31	3.29	6.12	7.09	4.14
Imipenem	0.35	0	6.12	6.10	9.31
Meropenem	4.5	—	0	38.46	48.57
Fosfomycin	—	—	0	—	0
Ciprofloxacin	22.37	12.84	19.05	27.03	33.79
Gentamicin	18.7	14.68	19.39	17.04	19.38
Piperacillin	—	—	—	—	—
Piperacillin/tazobactam	9.6	2.99	7.14	8.11	13.49
Cefoperazone/sulbactam	17.3	13.95	—	—	—
Ampicillin/sulbactam	41.2	—	24.21	29.15	30.74
Ceftazidime	19.98	15.13	19.73	18.24	23.10
Aztreonam	18.71	22.02	24.49	27.70	28.28

**Table 3:** Antibacterial drug usage between 2016 and 2020 (%).

Antibacterials	Years											
	2016		2017		2018		2019		2020		Total	
	DDDs	Rate (%)	DDDs	Rate (%)	DDDs	Rate (%)	DDDs	Rate (%)	DDDs	Rate (%)	DDDs	Rate (%)
*β*-Lactams	74879.0442	55.42	83786.48	58.05	89739.74	62.64	98187.65	62.17	72895.80	57.58	419488.72	59.31
Quinolones	21570.52	15.97	26223.50	18.17	24529.48	17.12	28977.33	18.35	23834.88	18.83	125135.72	17.69
Aminoglycosides	2279.4	1.69	2315.87	1.60	2157.93	1.51	2362.80	1.50	2167.93	1.71	11283.93	1.60
Tetracyclines	10	0.01	22.50	0.02	54.50	0.04	111.50	0.07	63.50	0.05	262.00	0.04
Carbapenem	1053.25	0.78	1039.50	0.72	892.25	0.62	1292.25	0.82	1720.50	1.36	5997.75	0.85
Macrolides antibiotics	19116.83	14.15	16929.00	11.73	12612.58	8.80	13897.84	8.80	12327.50	9.74	74883.76	10.59
Glycopeptides	194.25	0.14	266.25	0.18	385.00	0.27	348.75	0.22	312.75	0.25	1507.00	0.21
Lincomycin	7702.67	5.70	5846.33	4.05	5831.33	4.07	5801.33	3.67	5526.67	4.37	30708.33	4.34
Nitroimidazoles	5684.77	4.21	4989.63	3.46	4943.50	3.45	4225.17	2.68	5504.88	4.35	25347.95	3.58
Antifungals	2440.50	1.81	2970.25	1.93	1943.00	1.36	2469.00	1.56	1977.25	1.56	11620.00	1.64
Other	172.51	0.13	120.31	0.08	174.58	0.12	258.04	0.16	270.78	0.21	996.22	0.14

**Table 4:** Correlation between *Klebsiella pneumoniae* resistance rate and antimicrobial drug usage.

Resistance	DDDs								
	Β-Lactams	Quinolones	Aminoglycosides	Tetracyclines	Carbapenem	Macrolides antibiotics	Glycopeptides	Lincomycin	Nitroimidazoles
Amikacin	−0.987	−0.535	0.457	−0.573	−0.249	0.806	−0.238	−0.085	−0.724
Imipenem	−0.946	−0.871	0.824	−0.893	0.239	0.43	0.25	−0.547	−0.964
Meropenem	−0.971	−0.826	0.771	−0.851	0.154	0.506	0.166	−0.472	−0.938
Fosfomycin	0.809	0.1	−0.01	0.145	0.656	−0.986	0.648	−0.37	0.338
Ciprofloxacin	−0.021	0.732	−0.79	0.7	−0.998^*∗*^	0.73	−0.998^*∗*^	0.964	0.545
Gentamicin	−0.909	−0.917	0.877	−0.934	0.336	0.336	0.347	−0.629	−0.986
Piperacillin	−0.886	−0.244	0.156	−0.288	−0.54	0.951	−0.53	0.231	−0.471
Piperacillin/tazobactam	0.965^*∗*^	0.839	−0.786	0.863	−0.178	−0.486	−0.189	0.493	0.946
Cefoperazone /sulbactam	0.971^*∗*^	0.825	−0.771	0.85	−0.154	−0.507	−0.165	0.472	0.937
Ampicillin/sulbactam	0.872^*∗*^	0.946	−0.913	0.96	−0.411	−0.259	−0.422	0.69	0.996
Ceftazidime	0.124	−0.658	0.723	−0.623	0.865^*∗*^	−0.796	0.874^*∗*^	−0.931	−0.456
Aztreonam	0.352	0.933	−0.962	0.915	−0.901	0.423	−0.906	0.994	0.818

Note: the values in the table are *r* values (derived by the Pearson analysis in the SPSS software). ^*∗*^*P* < 0.05.

## Data Availability

All data generated or analyzed during this study are included within this article.
